# The Use of CT Coronary Angiography and CT Fractional Flow Reserve in the Investigation of Patients With Suspected Coronary Artery Disease

**DOI:** 10.7759/cureus.7908

**Published:** 2020-05-01

**Authors:** Mohammad Fawad Khattak, Sebastian Horne

**Affiliations:** 1 Cardiology, Russells Hall Hospital, Dudley, GBR

**Keywords:** coronary artery disease, ctca, ffr, angina, fractional flow reserve, coronary ct angiography, ischemic heart disease

## Abstract

Objective

To assess the diagnostic performance of CT fractional flow reserve (CT-FFR) and to assess whether its use in addition to CT coronary angiography (CTCA) changed the investigation and management of patients with suspected coronary artery disease (CAD).

Method

A retrospective case note review was carried out for 200 consecutive patients at Russells Hall Hospital, Dudley, United Kingdom, who had CTCA sent for Heartflow CT-FFR analysis (HeartFlow, Redwood City, CA) between January 2018 and December 2019.

Results

Patients with CT-FFR > 0.8 were significantly less likely to require further investigation with coronary angiography (p: < 0.00001) than those with CT-FFR < 0.8. The use of CT-FFR significantly reduced need for further functional imaging (6% vs 26%) (p: 0.00012). A total of 15 patients in this study had both a CT-FFR and an invasive FFR measured, with seven (46.66%) of the CT-FFRs correlating with the invasive FFR. Approximately 54% of patients who had a CT-FFR < 0.8 were found to have an invasive FFR of >0.8.

Of the 56 patients who underwent coronary angiography, the CT Coronary Artery Disease-Reporting and Data System (CAD-RADS) and angiography CAD-RADS were the same in 66% of the cases with 82% of CT CAD-RADS results being within ±1 of the angiography CAD-RADS.

Conclusion

The use of CT-FFR alongside CTCA led to a significant reduction in need for coronary angiography and functional testing. Further studies are required to look at the diagnostic accuracy of CT-FFR in direct comparison with invasive FFR.

## Introduction

Coronary artery disease (CAD) is a pathological process characterized by the accumulation of atherosclerotic plaques in the coronary arteries. It is the most common cause of death in the United Kingdom, and there are 80,000 annual deaths from CAD in the United Kingdom [1]. Therefore, appropriate diagnosis and treatment is important to improve prognosis in patients with CAD.

In 2016, the National Institute for Health and Care Excellence in the UK (NICE) recommended the use of CT coronary angiography (CTCA) as the first-line investigation of choice for patients with angina and no history of CAD [2].

CTCA has a high sensitivity and high negative predictive value for the diagnosis of CAD, but it does not determine whether these lesions significantly obstruct blood flow. Studies have shown that lesions that were initially considered severe on CTCA were ultimately found not to be hemodynamically significant in more than 50% of the cases [3]. This means that patients with significant stenosis on CTCA (>50%) will often require additional functional tests to identify lesion-specific ischemia [4].

Fractional flow reserve (FFR) measure during coronary angiography serves as the gold standard for identifying vessel-specific ischemia, with an FFR of <0.8 being used to identify significant flow-limiting disease. The Fractional Flow Reserve versus Angiography for Multivessel Evaluation 2 (FAME 2) trial showed that the use of FFR-guided percutaneous coronary intervention (PCI) led to better cardiovascular outcomes [5]. However, despite robust evidence supporting the of FFR and a recommendation from the European Society of Cardiology advocating its use in assessing hemodynamic benefit of intermediate grade stenosis, uptake of FFR has been low worldwide [6].

CT-FFR involves the use of anatomical models of the coronary vasculature imaged using CTCA and applying a mathematical model of coronary physiology and the subsequent use of computational models of fluid dynamics to estimate FFR.

HeartFlow (Redwood City, CA) has developed a software to produce CT-FFR results and has been FDA approved with NICE considering implementing it as part of the work-up for patients with suspected CAD [7,8].

The use of CT-FFR has numerous claimed benefits, including the ability to provide non-invasive functional assessments of lesions detected by CTCA without the use of any additional imaging, radiation or medication. NICE states that CT-FFR may have better diagnostic performance than CCTA alone or other functional tests and that its use may reduce the need for unnecessary invasive coronary angiography or other functional tests [8]. NICE believes that by adopting the use of CT-FFR the National Health Service (NHS) may be able to save a minimum of £9.1 million by 2022 through avoiding invasive investigation and treatment.

The aim of this study was to investigate the diagnostic performance of CT-FFR and whether its use in addition to CTCA changed the investigation and management of patients with suspected CAD at Russells Hall Hospital.

## Materials and methods

A retrospective case note review was carried out for 200 consecutive patients at Russells Hall Hospital, Dudley, United Kingdom, who had CTCA sent for HeartFlow analysis between January 2018 and December 2019.

Inclusion criteria were as follows: both male and female patients aged 18 years or above who had undergone CTCA of adequate quality to formally report on coronary anatomy. Patients who had CTCA for suspected acute coronary syndrome and those who did not have follow-up for cardiology were excluded from the study. Patients with contraindications for CTCA in the form of non-rate controlled atrial fibrillation, renal insufficiency (estimated glomerular filtration rate <30 mL/min/1.73 m^2^), possible pregnancy, and history of iodine contrast anaphylaxis were not included in the study.

CTCAs were performed with a 64-slice CT scanner, and the scans were prospective electrocardiogram-gated axial scans. If heart rate exceeded 80 beats/min, intravenous metoprolol was used five minutes before the scan. Iodine contrast material was used for the scan via a 18G or 20G intravenous cannula via a double-head power injector.

All the scans in this study were reviewed and reported by either consultant cardiologists or consultant radiologists with an interest in cardiovascular imaging. In each case, we calculated the CT Coronary Artery Disease-Reporting and Data System (CAD-RADS) score; looked at whether HeartFlow was able to generate a CT-FFR and noted this result using an FFR of <0.8 as a cut-off to determine hemodynamically significant stenosis; determined whether an invasive coronary angiogram and invasive FFR were performed, and whether any functional tests had been performed; and looked at medical outcomes after investigations.

All statistical analyses were performed using the SPSS Software for Windows, Version 21.0 (IBM Corp., Armonk, NY), with p < 0.05 considered statistically significant.

## Results

This observational study included a total of 200 patients, of which 123 (61.5%) were female. The mean age in this study was 63.4 ± 10.5 years. Approximately 98% of patients were found to have some evidence of CAD on CTCA, and 73% of patients had a CAD-RADS of 3 or higher signifying at least moderate (>50%) stenosis.

HeartFlow was able to generate a CT-FFR in 170 cases (85%). The CT-FFR was <0.8 in 29.4% of the cases. Fifteen patients in this study had both a CT-FFR and an invasive FFR measured, with seven (46.66%) of the CT-FFRs correlating with the invasive FFR. Approximately 54% of patients who had a CT-FFR <0.8 were found to have an invasive FFR of >0.8.

Coronary angiography was performed in only 10% of the patients with a CT-FFR >0.8 and 58% of the patients with a CT-FFR <0.8 demonstrating a statistically significant reduction in angiography when CT-FFR did not suggest a hemodynamically significant stenosis (p: <0.00001). Approximately 50% of patients whose HeartFlow was unable to generate a CT-FFR went on to have coronary angiography which is not statistically more than patients who had a CT-FFR generated (p: 0.3707). Figure 1 shows the proportion of patients who went on to have coronary angiography divided into the respective FFR results.

**Figure 1:** Did patients have angiogram after CTCA divided into groups depending on CT-FFR? CTCA, CT coronary angiography; FFR, fractional flow reserve.

Patients with a CT-FFR generated had a significant reduction (6% vs 26%) (p: 0.00012) in need for further functional tests when compared to patients with no CT-FFR available. Figure 2 demonstrates the different tests used after CTCA.

**Figure 2:** Investigations used after CTCA. CMRI, cardiac MRI; DSE, dobutamine stress echocardiography; ETT, exercise tolerance test; MPI, myocardial perfusion imaging.

Of the 56 patients who underwent coronary angiography, the CT CAD-RADS and angiography CAD-RADS were the same in 66% of the cases with 82% of CT CAD-RADS results being within ±1 of the angiography CAD-RADS. These results are illustrated in Figure 3.

**Figure 3:** Comparing the CAD-RADS result from CTCA with CAD-RADS result from coronary angiography. CAD-RADS, Coronary Artery Disease-Reporting and Data System; CTCA, CT coronary angiography.

In terms of medical outcomes, the vast majority of patients were medically managed with optimal drug therapy (82%). A total of 29 patients (14.5%) went on to have PCI and seven patients (4.5%) went to have coronary artery bypass surgery. Figure 4 illustrates these outcomes.

**Figure 4:** Outcomes after investigation. CABG, coronary artery bypass graft surgery; OMT, optimal medical therapy; OMT-for review RE PCI, patients who have follow-up to assess for response after OMT-plan for PCI if still symptomatic; PCI, percutaneous coronary intervention.

## Discussion

In this retrospective study, our results have demonstrated that the use of CT-FFR had significantly reduced the need for coronary angiography in patients with CT-FFR > 0.8 and also reduced the need for further functional investigations when compared to CTCA alone. CTCA when compared to coronary angiography was able to generate results with similar CAD-RADS in the vast majority of patients.

When comparing CT-FFR with invasive FFR, we found that more than 50% of the patients with a CT-FFR of <0.8 went on to have a normal invasive FFR. Given the low number of patients with both CT-FFR and invasive FFR, larger studies will be required in the future to better assess and comment on accuracy of CT-FFR in comparison to invasive FFR.

Invasive FFR uptake remains low due to costs associated with it, time added to coronary angiography, patient discomfort to hyperemic stimulus, and contraindications to adenosine use. The use of CT-FFR is an attractive prospect as its use allows both anatomical and functional assessment of coronary arteries without any further imaging/radiation or use of medications. This will allow departments to reduce costs by reducing the amount of invasive angiography performed. The reduction in invasive procedures will also free up resources both in terms of staff and equipment.

A recent retrospective Japanese trial comparing invasive FFR and CT-FFR in 47 patients found that CT-FFR had high diagnostic accuracy for detecting hemodynamically significant CAD and served as an effective gatekeeper to decide which patients required invasive angiography [9]. Further larger studies are required to look specifically at patients who have both invasive FFR and CT-FFR to allow further study in the diagnostic accuracy of CT-FFR and to help determine whether CT-FFR should be combined with CTCA as a first-line investigation in the assessment of patients with suspected CAD.

## Conclusions

The use of CT-FFR alongside CTCA led to a significant reduction in need for coronary angiography and functional testing. Further studies are required to look at the diagnostic accuracy of CT-FFR in comparison to invasive FFR.
